The article "Human sperm degradation of zona pellucida proteins contributes to fertilization" was published in 2015. Journal: Reprod Biol Endocrinol.

# Human sperm degradation of zona pellucida proteins contributes to fertilization

**DOI:** 10.1186/s12958-015-0094-0

**Published:** 2015-09-02

**Authors:** Analilia Saldívar-Hernández, María E. González-González, Ana Sánchez-Tusié, Israel Maldonado-Rosas, Pablo López, Claudia L. Treviño, Fernando Larrea, Mayel Chirinos

**Affiliations:** Departamento de Biología de la Reproducción, Instituto Nacional de Ciencias Médicas y Nutrición Salvador Zubirán, México, D.F. 14080 Mexico; Departamento de Genética del Desarrollo y Fisiología Molecular, Instituto de Biotecnología, UNAM, Cuernavaca, 62210 Mexico; Instituto Mexicano de Alta Tecnología Reproductiva (Inmater), Mexico, D.F. 11000 Mexico

**Keywords:** Human sperm, Zona pellucida, ZP penetration, Fertilization

## Abstract

**Background:**

The mammalian oocyte extracellular matrix known as the zona pellucida (ZP) acts as a barrier to accomplish sperm fusion with the female gamete. Although penetration of the ZP is a limiting event to achieve fertilization, this is one of the least comprehended stages of gamete interaction. Even though previous studies suggest that proteases of sperm origin contribute to facilitate the passage of sperm through the ZP, in human this process is not yet fully understood. The aim of this study was to determine the ability of human sperm to degrade recombinant human ZP (rhZPs) proteins and to characterize the proteases involved in this process.

**Methods:**

Purified rhZP2, rhZP3 and rhZP4 proteins were incubated with capacitated sperm and the proteolytic activity was determined by Western blot analysis. To further characterize the proteases involved, parallel incubations were performed in the presence of the protease inhibitors o-phenanthroline, benzamidine and MG-132 meant to block the activity of metalloproteases, serine proteases and the proteasome, respectively. Additionally, protease inhibitors effect on sperm-ZP binding was evaluated by hemizona assay.

**Results:**

The results showed that rhZPs were hydrolyzed in the presence of capacitated sperm. O-phenanthroline inhibited the degradation of rhZP3, MG-132 inhibited the degradation of rhZP4 and benzamidine inhibited the degradation of the three proteins under investigation. Moreover, hemizona assays demonstrated that sperm proteasome inhibition impairs sperm interaction with human native ZP.

**Conclusions:**

This study suggests that sperm proteasomes could participate in the degradation of ZP, particularly of the ZP4 protein. Besides, metalloproteases may be involved in specific degradation of ZP3 while serine proteases may contribute to unspecific degradation of the ZP. These findings suggest that localized degradation of ZP proteins by sperm is probably involved in ZP penetration and may be of help in understanding the mechanisms of fertilization in humans.

## Background

During mammalian fertilization, sperm should be able to reach the cumulus-oocyte complex, get through the hyaluronic matrix of the cumulus and penetrate the zona pellucida (ZP) in order to fuse with the egg. Despite the limiting nature of the last step, the underlying mechanisms that mediate the ZP penetration are barely understood. During the female tract transit, spermatozoa undergo a series of biochemical and functional changes, known as capacitation [1], that prepare the cells for an ultimate exocytosis event called acrosome reaction. This event allows the release of molecules from the acrosome -such as proteases- in the surroundings of the ZP. Human ZP is mostly constituted by four glycoproteins, named ZP1, ZP2, ZP3 and ZP4, being the ZP1 the least abundant [2]. Mechanical force applied by the capacitated spermatozoa in motion is essential to penetrate the ZP but the physical force generated by the flagellum may not be sufficient to enable sperm to push through this matrix [3]. There is growing evidence that sperm proteases may play a relevant role during gamete interaction [4] and that some extent of ZP protein degradation occurs during sperm-ZP penetration [5]. Besides, sperm proteases involved in penetration are likely to be located either in the surface of the plasma membrane or in the acrosome, since during penetration spermatozoa remain associated to ZP components by receptors located in the inner acrosomal membrane.

Proteolytic hydrolysis of ZP could be mediated by acrosomal/membrane associated proteases or by the controlled degradation of the ubiquitin-proteasome system. Evidence of these two protein degradation systems have been widely described in sperm of several species. In mouse, the most plausible candidates to be involved in ZP degradation are the serine protease TESP5 and the proteasome while acrosin, another serine protease, could also play an indirect role by dispersing acrosomal matrix content during acrosome reaction [reviewed by [4]]. However, the ZP degradation mechanism may not be conserved in all mammals. Indeed, while proteasome inhibitors block ZP penetration in porcine [5, 6], some studies suggest that bull sperm get use of matrix metalloprotease 2 (MMP2) and acrosin to accomplish ZP digestion during penetration [7]. Regarding human sperm, several proteases have been identified in the acrosome, such as acrosin and MMP2 and MMP9 (metalloproteases) [8, 7]. The proteasome is also present in human sperm located in the head, middle piece [9, 10] and the surface on spermatozoa [11]. Different investigations have demonstrated proteasome participation during human sperm capacitation [12], acrosome reaction [13, 14] and ZP binding [15], but its contribution during ZP penetration remains unknown. If a proteasome dependent ZP degradation occurs during penetration, ZP protein/proteins are then likely to be ubiquitinated, either by a maturation process during oogenesis (as in the pig) [6] or by a sperm extracellular machinery (as in ascidians) [16], but ZP proteins ubiquitination in human has not been properly investigated.

All the evidence collected up to date indicates that sperm proteases may be involved in human sperm penetration of ZP but this process remains unestablished due to the limited access to native human ZP. In the present study, we show evidence that human and mouse ZP were ubiquitinated and that human sperm is able to degrade recombinant human ZP proteins by a proteolytic-mediated process. In addition, proteasome inhibition reduced sperm binding to human native ZP. Therefore, results herein presented indicate that sperm proteases participate in the mechanism of ZP penetration during fertilization.

## Methods

All procedures herein described were undergone after protocol approval by the Institutional Review Board (IRB; Comité de Ética en Investigación) from the Instituto Nacional de Ciencias Médicas y Nutrición Salvador Zubirán, approved on 02/27/2012 with the reference number 564. The experimental procedures were executed between March 2012 and March 2014. IRB also approved the informed consent read and signed by each participant in the study.

### Zona pellucida immunofluorescence

The presence of ubiquitin (Ub) conjugates in human zona pellucida was investigated by immunofluorescence of post-mortem ovary tissues and mature oocytes. Ovary tissues were formalin fixed and paraffin embedded in order to perform 5–8 μm slices of the tissue. Afterwards, consecutive tissue sections were deparaffinized, rehydrated and blocked for 1 h with 3 % bovine serum albumin in phosphate buffered saline (PBS) for overnight incubation with rabbit anti-Ub antibody (Kamiya Biomedical Co., Seattle, WA) or with a rabbit immune serum against Heat-Solubilized Pig ZP (anti-HSPZ) that recognizes human native as well as recombinant ZP proteins [17]. After 3 washes with PBS, specimens were incubated for 1 h with a goat anti-rIgG antibody coupled to Cy3. Slides were again washed with PBS, mounted with Vectashield (Vector Laboratories) and samples were simultaneously examined by fluorescence and phase-contrast microscopy. On the other hand, cumulus-free mature oocytes from women under ovarian stimulation treatment for assisted reproduction techniques were employed for immunofluorescence analysis and preserved frozen in liquid nitrogen until use. After defrosting, they were fixed with 4 % p-formaldehyde for 30 min at room temperature, processed following the procedure above described and analyzed by confocal fluorescence microscopy (Zeiss, Weimar, Germany). Fresh oocytes from hyperstimulated mouse were also analyzed by immunofluorescence as positive controls. In all cases, negative control specimens were obtained by incubation with either total gamma globulin from rabbit or in the absence of primary antibodies but otherwise processed as test slides.

### Preparation of rhZP2, rhZP3 and rhZP4 proteins

The cDNAs coding for human ZP2, ZP3 and ZP4 were expressed in Sf9 cell line as previously described [18, 19]. Recombinant viruses containing the different protein sequences and a 6xHis tag were used for infection of the cell line in TNM-FH medium containing 10 % fetal bovine serum (Pharmingen, San Diego, CA) at 27 °C and cultured for 4–5 days. Before harvesting, Sf9 cells were subjected to heat-shock conditions to enhance the production of ubiquitin conjugates by incubation at 41 °C for 30 min followed by a 3 h recovery period at 27 °C. Afterwards cells were harvested and used for affinity protein purification using Ni-NTA agarose beads (Invitrogen, Carlsbad, CA) under denaturing conditions. After renaturing by a decreasing urea gradient, purified proteins were used for experiments here described either attached to the agarose beads or in solution after elution from the resin with 100 mM imidazole.

### Characterization of purified rhZP proteins

Purified rhZP proteins were characterized by SDS-PAGE on 10 % polyacrylamide gels and either stained with Coomassie brilliant blue (CBB) or blotted onto nitrocellulose membranes to be analyzed by Western Blot. Identical membranes were probed with anti-HSPZ serum and the rabbit anti-Ub antibody. Antibody detection was undergone by incubation with protein A coupled to ^125^I, followed by autoradiography.

### Sperm samples collection and preparation

Human semen samples used in this study were obtained by masturbation from healthy normozoospermic donors after 3–5 days of sexual abstinence. Ejaculates were assessed and processed using standard methods [20]. For capacitation, samples were centrifuged through a discontinuous density gradient (Isolate; Irvine Scientific, Santa Ana, CA), and resulting pellets were incubated overnight at 4 °C with equal volumes of Modified Sperm Washing Medium (MSWM, Irvine Scientific) and Refrigeration Test Yolk Buffer (Irvine Scientific). After washing with MSWM, sperm pellets were overlaid with 1.2 ml of modified Human Tubal Fluid medium (HTF; Irvine Scientific) supplemented with 0.3 % human serum albumin and 1 mM sodium pyruvate (supHTF) for *swim-up* separation, by incubating for 1 h at 37 °C in 5 % CO_2_ and 95 % of humidity with the tube inclined at a 45° angle. The uppermost layer (1.0 ml) with the motile sperm fraction were recovered and incubated for 4 h at 37 °C before their use for experiments.

### Sperm function analysis

Protease inhibitors were used to characterize the participation of sperm proteases in rhZP proteins degradation. For this purpose, protease inhibitors effects on sperm viability, motility, spontaneous acrosome reaction (AR) and calcium ionophore (CaI) induced AR were evaluated, following methodologies previously described [18]. The protease inhibitors selected and evaluated were MG-132 for proteasome mediated degradation, o-phenanthroline for metalloproteases and benzamidine for serine proteases. Concentration ranges tested for each protease inhibitor were selected according to previous studies [6, 21, 22]. After capacitation, sperm aliquots were incubated with the protease inhibitors at different concentrations or corresponding vehicles during 30 min and sperm variables were evaluated. Viability was evaluated by staining with the trypan blue vital exclusion dye followed by analysis under the microscope to determine the percentage of live cells. Motility changes were analyzed by phase contrast microscopy and sperm movement was graded following W.H.O. motility criteria [20]; after evaluating at least 200 cells per treatment, data were presented as percentage of sperm with progressive motility (a + b), non-progressive motility (c) and immotility (d). Spontaneous and CaI (A23187 10 μM, Sigma) induced AR were evaluated after sperm fixation with 70 % ethanol followed by acrosome staining the PSA lectin coupled to FITC [18]. Each experiment was repeated at least three times. Values are presented as the mean ± SEM and treatments groups were analyzed using the GraphPad Prism 5.01 software (GraphPad, San Diego, CA, USA), using one way ANOVA and Tukey’s multicomparison for post hoc test, considering significant a *P* value ≤ 0.05.

### Evaluation of sperm mediated rhZPs degradation

Experiments were carried out using sperm aliquots from a single semen sample for simultaneous analysis of rhZP2, rhZP3 and rhZP4 degradation. Agarose beads immobilized rhZPs were incubated in 48-well plates with 2x10^6^ capacitated sperm in supHTF medium for 16 h at 37 °C in 5 % CO_2_ and 95 % of humidity, in the presence or absence of protease inhibitors. At the end of incubation, sperm motility was checked under the microscope and experiments with total motility below 70 % were discarded. Agarose beads were gently washed twice with PBS and mixed with Laemmli denaturing sample buffer. All samples were used for SDS-PAGE and analyzed by Western blot using anti-HSPZ as primary antibody. When protease inhibitors were used, capacitated sperm were pre-incubated for 30 min with the inhibitors before addition to the agarose immobilized rhZPs. Degradation experiments were repeated at least 5 times. Densitometry analyses were performed using the ImageJ software.

### Hemizona assay

Human oocytes from women undergoing ovulation induction for assisted fertilization procedures were employed for hemizona assays (HZA) [23]. Only non-viable oocytes (either immature oocytes that were not inseminated or mature oocytes that failed to be fertilized by conventional ICSI) were collected and stored at 4 °C in 20 mM Tris–HCl (pH 7.2-7.6), 2 M (NH_4_)_2_SO_4_ and 0.5 % dextran until use. On the day of the experiment, oocytes were thoroughly washed with HTF medium before bisection with a microscalpel attached to micromanipulators (Narishigue, Tokyo, Japan) to separate ZPs from oocytes and cut them into equal halves (hemizonas, HZ). HZs were transferred to 50 μl drops of supHTP under mineral oil and 3–5 x 10^4^ capacitated sperm in 50 μl of supHTF were added to each drop for co-incubation for 4 h at 37 °C in an atmosphere of 5 % CO_2_. For each HZA, sperm aliquots were pre-incubated for 30 min with either the protease inhibitor at twice the final concentration chosen for the assay or the corresponding vehicle in supHTF before addition to matching counterparts. At the end of the co-incubations, HZ were removed and washed by repeated vigorous pipetting and the number of sperm tightly bound to the outer surface of each HZ was determined under the microscope. Results of the HZA were expressed as the HemiZona Index (HZI = [number of test sperm bound/number of control sperm bound] × 100) [24]. At least three independent experiments were performed using sperm samples from different donors. Data are expressed as mean ± SD. The different groups of HZA were compared by the paired sample *t*-test.

## Results

### Ubiquitination of native zona pellucida at different stages of oocyte maturation

The presence of ubiquitin (Ub) in human oocytes was investigated by indirect immunofluorescence analysis using consecutive slices of ovary tissue. In Fig. 1, positive labeling for ZP is shown when incubated in the presence of anti-HSPZ (Fig. 1a) whereas no signal was detected in the oocytes of negative control (Fig. 1b). When ovary sections were incubated with anti-Ub antibodies, positive staining was only detected inside oocytes as well as in granulosa cells, suggesting that most of the oocytes in the studied specimens were probably under follicular atresia (Fig. 1c and d). In order to investigate whether ZP proteins ubiquitination appears later during follicle development, we studied ubiquitination in more mature oocytes recovered after ovarian stimulation. Under this condition, a ZP positive signal was detected in the presence of the anti-HSPZ serum (Fig. 2a). Incubation with anti-Ub antibodies showed positive staining in the ZP as well as in the oocyte plasma membrane (Fig. 2b), suggesting that ZP protein/proteins ubiquitination appears at advanced stages of oocyte development. Control incubations in the absence of primary antibody showed no fluorescent signal (Fig. 2c). Furthermore, the specificity of the Ub recognition was demonstrated by competence experiments where saturation of anti-Ub antibody with free Ub visibly reduced the immunofluorescent signal (Fig. 2d). Mouse oocytes from hyperstimulated females were also employed as controls for antibody specificity, where ZP ubiquitination was also detected while virtually no signal was observed in the oocyte (Fig. 2e).

**Fig. 1:** Presence of ubiquitin in human ovary tissue. Immunofluorescent analysis of formalin fixed ovary sections, using for primary detection either anti zona pellucida serum (anti-HZPZ) (**a**), total gamma globulins from rabbit (**b**) or anti-Ub antibodies (**c** and **d**). Afterwards, all slices where incubated with secondary antibody and mounted for examination using phase-contrast (*left panels*) or epifluorescence (*right panels*). Ub was mostly detected inside oocytes and no signal was detected in the ZP (*indicated with white arrows*) of oocytes from early or developed follicles. Original magnification x400

**Fig. 2:** Assessment of ubiquitin in mature oocytes. *Left panel* shows phase-contrast images of analyzed oocytes, *center panel* displays the corresponding confocal fluorescent images with pseudocolor and *right panel* the merged images of the phase-contrast image and the fluorescence image. Human oocytes discarded from assisted reproduction techniques were collected and kept frozen until use for immunofluorescence studies for detection of (**a**) ZP; (**b**) Ub; (**c**) No primary detection (negative control without primary antibody); (**d**) Antibody competence (Anti-Ub antibodies + Ub protein). (**e**) Mouse oocytes obtained from hyperstimulated females were used as positive control by incubating with anti-Ub as positive control. Specific staining for Ub was detected in the ZP of both species

### Production of ubiquitinated rhZP proteins

Considering that human native ZP proteins from mature oocytes are ubiquitinated, we produced rhZP2, rhZP3 and rhZP4 proteins as well as their ubiquitinated forms by the use of an expression system that allows the production of proteins with post-translational modifications, as described in Materials and Methods. This procedure allowed us to obtain highly enriched purified rhZP proteins (Fig. 3a). When these purified proteins were tested with the anti-HSPZ serum, proteins with the expected molecular weights for ZP2 (80 kDa), ZP3 (55 and 65 kDa) and ZP4 (66 kDa) were detected [19], besides some additional protein bands of higher and lower molecular weight (Fig. 3b). Western blots of rhZP proteins with anti-Ub revealed that at least some of the high molecular weight forms of the proteins were ubiquitinated (Fig. 3c). In addition, few low molecular weight proteins were also detected by the anti-Ub antibody which may correspond to Ub-targeted ZP proteins already involved in the proteasome degradation system of the Sf9 cells or to unspecific degradation products. The overall results indicate that the baculovirus expression system used in this study was able to produce ZP proteins conjugated to Ub moieties.

**Fig. 3:** Obtaining of ubiquitinated recombinant human ZP proteins. Human ZP2, ZP3 and ZP4 proteins were expressed in Sf9 cell line under heat shock conditions followed by affinity purification. (**a**) The purity of rhZP proteins was examined by SDS-PAGE followed by staining with CBB. (**b**) The identity of purified proteins was determined by Western blot using anti-HSPZ for primary detection. (**c**) Ubiquitination levels of purified rhZP proteins were assessed by Western blot of same proteins using anti-Ub antibodies

### rhZPs proteins degradation by capacitated sperm

Sperm ability to perform proteolytic activity on rhZPs was investigated by the co-incubation of capacitated spermatozoa with the recombinant proteins, followed by Western blot with the anti-HSPZ serum to detect molecular weight changes in rhZPs. Figure 4 shows that incubations with capacitated sperm caused a reduction in the abundance of the three rhZP protein bands at their corresponding full length molecular weights (black arrows). Correspondingly, rh ZP2 and rh ZP4 abundance reductions were accompanied by the appearance of a novel protein band pattern of lower molecular weight. Control incubations of rhZPs in the absence of capacitated spermatozoa resulted in no changes in the molecular weight patterns and spermatozoa alone showed no signal, demonstrating the specificity of the anti-HSPZ serum. This approach suggested that capacitated human sperm is able to degrade rhZP proteins.

**Fig. 4:** Sperm degradation of rhZP proteins. Agarose beads immobilized rhZP2, rhZP3 and rhZP4 proteins were co-incubated under capacitating conditions with human spermatozoa for 16 h. Afterwards, beads were washed and bound proteins were solubilized in Laemmli denaturing sample buffer for Western blot analysis with anti-HSPZ. Control incubations without rhZP proteins and without sperm are also presented. *Black arrows* indicate the expected full length for each rhZP protein. Spm = spermatozoa

### Protease inhibitors prevent rhZPs degradation

To evaluate the specific activity of human sperm proteolytical activity on rhZPs, protease inhibitors were employed. However, they were previously tested in order to determine if they could affect sperm function variables related to sperm fertilization ability, such as viability, motility and acrosome reaction (AR). When we analyzed the effects of the protease inhibitors MG-132, o-phenanthroline and benzamidine on sperm function, we found no effect on motility parameters (Fig. 5a) as well as on spontaneous and CaI induced AR (Fig. 5b). Moreover, no significant changes in sperm viability were detected with any of the treatments, since live sperm values were above 95 % under all tested conditions.

**Fig. 5:** Effects of protease inhibitors on sperm function. (**a**) Effects on motility: Percentages of progressive motility (*dark grey bars*), non-progressive motility (*white bars*) and immotility (*light grey bars*) after sperm incubation in the presence of MG-132, O-phenanthroline and benzamidine. (**b**) Effects on acrosome reaction: Percentage of spontaneous (*grey bars*) and calcium ionophore (*CaI*) induced (*black bars*) acrosome reaction of sperm treated with MG-132, O-phenanthroline and benzamidine. Acrosomal status was evaluated after staining with FITC-PSA and percentage of reacted cells were determined. Values in percentage are presented as the mean ± SEM. No significant differences between controls (in the absence of inhibitors) and treatments were detected. N ≥ 3 experiments

Sperm co-incubations with immobilized rhZP2, 3 and 4 were carried out in the presence of MG-132, o-phenanthroline and benzamidine to characterize proteases participation in rhZPs degradation. Representative Western blots with anti-HSPZ (Fig. 6, left panel) are presented accompanied by corresponding histogram densitometry analyses (Fig. 6, right panel) for enhanced detection of molecular masses changes and protein abundance. As expected, sperm-rhZPs incubations in the absence of inhibitors showed decrease in full length rhZPs (see black arrows) accompanied by increase in low molecular weight forms of each rhZP (see brackets). No changes in the degradation protein pattern was observed when rhZP2 was co-incubated with sperm in the presence of MG-132 and o-phenanthroline, but benzamidine partially preserved the integrity of rhZP2 suggesting that some of the observed sperm proteolysis of rhZP2 was mediated by serine proteases. Likewise, the proteolysis of rhZP3 was prevented in the presence of benzamidine and also with o-phenanthroline, suggesting that serine proteases as well as metalloproteases may be involved in rhZP3 degradation, while MG-132 showed no effect in the overall proteolysis of this protein. Regarding rhZP4 degradation, it was inhibited by benzamidine and MG-132 and not by o-phenanthroline, denoting that sperm proteasomes and serine proteases could mediate the degradation of this protein.

**Fig. 6:** Differential degradation of rhZP2, rhZP3 and rhZP4 proteins by capacitated sperm. Agarose beads immobilized rhZP proteins were incubated in the absence or presence of capacitated sperm with and without protease inhibitors, and analyzed by Western blot with anti-HSPZ. *Left panel* shows representative Western blots for sperm degradation of rhZP2, rhZP3 and rhZP4. *Right panel* presents corresponding densitometry histograms, showing the effects of MG-132, o-phenanthroline and benzamidine over the rhZPs protein degradation patterns. *Black arrows* indicate proteins at the expected full length size and *brackets highlight* low molecular weight forms of each protein

### Proteasome inhibitor reduces sperm-ZP binding

To further investigate if sperm mediated rhZP proteins degradation is comparable to what physiologically occurs during gamete interaction, HZA were performed in the presence of the protease inhibitors under investigation. As shown in Fig. 7, only MG-132 was able to reduce the index of sperm tightly bound to the ZP. This result suggests that under physiological conditions proteasome activity may contribute during the sperm binding/penetration of the ZP.

**Fig. 7:** Effect of protease inhibitors on sperm binding to human native zona pellucida. Protease inhibitors effects on sperm-ZP binding were investigated by hemizona assay as described in Materials and Methods. For each hemizona incubated in the presence of a protease inhibitor, the matching counterpart was incubated with medium. HZI were estimated and presented as percentage (Mean ± SD). *N* = 4. (*) Control and treatment were significantly different, *p* = 0.0002

## Discussion

Since early studies on fertilization, a possible role of sperm proteases during mammal ZP penetration has been suggested due to the evident physical limitation that this extracellular matrix impose to sperm fusing with the oocyte. The presence of serine proteases and metalloproteases in human sperm has been widely documented but their participation during the ZP recognition/penetration step remains unclear. However, several reports, mostly performed in non-human mammal models, suggest that they may contribute to this process. In the human, information on this issue is limited particularly due to difficulties in the access to human native ZP for research. By use of bioactive recombinant human ZP proteins, this work demonstrate that human capacitated sperm are able to degrade rhZP2, rhZP3 and rhZP4, and that such proteolytic activity is partially prevented by different protease inhibitors. Particularly, benzamidine, a serine-protease inhibitor, was able to reduce the proteolysis of rhZPs. Acrosin, a serine-protease localized in the acrosomal matrix, is the most abundant protease in human sperm and has been the target of many investigations about its role in fertilization. Its localization supports a possible participation during ZP penetration, since only acrosome reacted spermatozoa penetrate the ZP. In this regard, the observation that recombinant human proacrosin/acrosin binds to rhZP2 [25] and the presence of acrosin antibodies in sera from infertile women [26] supports the participation of acrosin in the process of fertilization. However acrosin knockout mice have revealed that it is not essential to fertilize the oocyte [27], suggesting that, in addition to it, another proteases may be involved in this process. In this regard, metalloproteases are a family of proteolytic enzymes that degrade protein components of the extracellular matrix, so we studied the effect of an inhibitor of these enzymes on sperm-induced breakdown of rhZPs. The results in this study showing that o-phenanthroline affected the ability of sperm to degrade rhZP3 might represent another mechanism by which sperm penetrate the ZP. As far as we know, no previous evidence has suggested a possible role for human sperm metalloproteases during interaction with the ZP. Nevertheless, clinical observations have previously described that normal and abnormal semen samples have different metalloproteases profile [8], suggesting a correlation between metalloproteases and sperm fertilization capacity.

On the other hand, in recent years the presence of proteasomes in human [13, 9] and other mammalian [28] spermatozoa has been reported and consequently their participation in sperm ZP penetration has also been subject to investigations. In porcine, it has been demonstrated that proteasomal interference prevents zona pellucida penetration and fertilization [6] and that sperm proteasome degrades the ZP, specifically the ZPC protein that is homologue to human ZP3 [5]. If a proteasome proteolysis of ZP occurs during penetration of this oocyte vest, ubiquitination of ZP proteins could be expected. To address this hypothesis, we explored if native human ZP proteins were ubiquitinated and found that ZP appears to be ubiquitinated but only in mature oocytes. Attempts to detect ubiquitin on ZP from early stages oocytes were not successful, suggesting that either ZP proteins were not ubiquitinated or that the degree of ubiquitination was lower than the detection limit of the immunofluorescence technique employed in this study. Instead, we observed ubiquitination in oocytes as well as granulosa cells in primordial, primary and secondary follicles, a finding that may be of biological relevance since this process is associated with oocyte resorption, a process normally occurring during the menstrual cycle. Indeed, ubiquitination is thought to be part of the mechanisms by which follicles are destined for atresia [29].

There are several observations that suggest and support that proteasome may control sperm capacitation and in turn have an indirect effect on sperm capability to bind and penetrate the ZP. For instance, proteasomal inhibition reduced the protein Ser-phosphorylation that accompanies sperm capacitation [26]. However, the proteasome may also have a direct participation during sperm-ZP interaction. As we employed already capacitated sperm for incubation with rhZPs in the presence of the proteasomal inhibitor MG-132, our results indicate that a compromised proteasome function lead to a reduced sperm capacity to degrade rhZP4. Furthermore, proteasomal participation in sperm-ZP interaction was confirmed for native human ZP in hemizona assays. However, the participation of sperm serine proteases and metalloproteases during ZP binding could not be confirmed with this approach, but the functional and mechanistic redundancy widely described for gametes during mammalian fertilization [30] may be masking the participation of these proteases in sperm-ZP interaction in this approach.

## Conclusions

In summary, in this study we present evidence that capacitated sperm are able to degrade rhZP proteins, suggesting the presence of a sperm-dependent proteolysis mechanism that may participate in the process of sperm interaction and penetration of the ZP. Moreover, we suggest that an ubiquitin proteasome pathway is required for the targeted degradation of human ZP proteins. Therefore these results may contribute to the understanding of the molecular mechanisms involved in the process of gamete interaction during human fertilization.
